# Research on the Design of Intelligent Music Teaching System Based on Virtual Reality Technology

**DOI:** 10.1155/2022/7832306

**Published:** 2022-04-07

**Authors:** Wei Chen

**Affiliations:** Music and Dance Department, Zhengzhou Normal University, Zhengzhou 450000, Henan, China

## Abstract

With the continuous development and innovation of artificial intelligence technology, its application in the field of music education is also increasing, music classroom has accepted and applied a more efficient and intelligent teaching system. In the reform of teaching, virtual reality (VR) technology has gradually become a new means which occupies a place in the field of education and scientific research. The teaching system based on virtual reality has been focused in all kinds of teaching. Therefore, in this paper, VR is used to build a music teaching system based on model embedding, bread capture, packing capture and camera establishment, so as to implement the music teaching platform based on VR. Through the construction of different virtual elements, it can better achieve the goals of public participation and can effectively stimulate the singer's sensory organs.

## 1. Introduction

Virtual Reality (VR) technology and augmented reality (AR) technology attract more and more people to engage in the research and development of related theories and technologies [1]. At present, VR technology and AR technology are widely used in entertainment [2], tourism, medical [3], games [4], education [5], etc. Many VR and AR companies and related talents [6] have emerged in the society. Many colleges and universities are naturally unwilling to fall behind. They have built a series of virtual laboratories and virtual courses [7] related to virtual reality and augmented reality. Moreover, not only higher education institutions, but also many training institutions have seized the opportunity, a lot of courses about virtual reality are set up to continuously import talents for the society [8].

In the reform of teaching, the education mode has gradually changed from the traditional blackboard-writing and PPT teaching to the combination of informatization and traditional education [9]. Especially in the field of practice teaching in higher education, According to “The Implementation Plan for Accelerating the Modernization of Education (2018–2022)” issued by the general office of the CPC Central Committee and the general office of the State Council, it is mentioned that “efforts should be made to build new education and teaching mode based on information technology,” “it is necessary to develop the construction of national teaching project about virtual simulation experiment,” which points out that we should make full use of computer simulation technology to carry out the construction of virtual simulation experiment teaching, promote the sharing of advantageous educational resources in Colleges and universities, solve the problem of unreasonable allocation of educational resources, and improve the overall level of education in China [10, 11].

## 2. Analysis of Virtual Reality Technology

### 2.1. Virtual-Real Integration Technology

As an important basis to distinguish VR and AR technology, Virtual-real integration technology is one of the three characteristics of augmented reality technology. The “real” here refers to the real objects captured by the camera, and the “virtual“ here is composed of models, sounds and words created by computer software, which is a supplement to the objects in real world. Then, virtual real integration technology is used to stack the virtual thing and the reality to ensure the consistency of illumination, geometry and motion, so as to realize seamless superposition and achieve augmented reality [12, 13].

Virtual-real integration technology is realized by three methods: 3D model reading and rendering, pixel operation and texture rendering. The main principle of texture rendering is to take the real image as the texture data, and then regard the texture as the unit to draw the real image on the surface perpendicular to the virtual camera, afterwards, a virtual object is generated between its plane and the camera [14]; the basic principle of pixel operation is to use its function to read the data of the real image into the cache and draw the virtual object; In addition, 3D model reading and drawing is mainly through reading the format of the 3D model, and then reading the data (vertex and face of the model); Furthermore, open GL can draw objects through these data and materials [15]. The way of reading the data of 3DS model is employed to realize the integration of virtual information and landmarks.

An experiment in VR course on music genre recognition was carried out in a primary school, which immerses students in different musical styles (such as classical, country, jazz and swing) through mobile VR devices. The results show that compared with the traditional courses of printed materials and passive listening, the combination of mobile VR technology and traditional teaching methods can improve experience of music learning in the aspects of actively listen, attention focusing and others [16]. The combination of VR technology and these related courses can better solve the disadvantages in the traditional teaching process. Through VR teaching, the scene can be vividly presented in front of the students. While students will not be limited by time, frequency, distance, safety and other factors. VR equipment can be used to listen to the sound repeatedly, so as to achieve emotional integration, which can not only enhance the interest in class but also solve the practical problems in music teaching.

### 2.2. Unity3d Technology

Unity3d is a multi-platform game tool designed to be easy to use from the beginning [17]. As a fully integrated professional application, it is also a powerful game engine with multi-million dollar, as well as a fully integrated editor [17].

Unity3d and integrated development environment are perfectly combined [18]. This joint integration allows the editor to do whatever it takes to publish a game [18]. Simple, visual, intuitive, these features of editor make the construction of games more interesting. Originally a game development kit for Mac, windows, and Linux, it was developed to be deployed on iPhone and Wii, or on the web [19]. However, this is not common in game engines that Unity3d is a scripting language. Another example is that Second Life also uses mono as the script engine and C# as the scripting language [20]. Its application in the game engine promoted the progress of Mono itself, including Mono.Simd, which makes Mono or managed code more suitable for the development of game [21].

## 3. Classifications of Music Teaching System Based on Virtual Reality Technology

### 3.1. Model Embedding System

In virtual reality, model embedding system is an important factor to express the effect of experience, and its function of geometric segmentation plays a decisive role in the fluency of experience in scene interaction. The same model is divided into three levels of LOD (levels of detail) accuracy specifications, so as to flexibly switch the model accuracy in different Line-of-sight range [22, 23]. The principle that this switching mode must follow is to ensure that the model accuracy of the foreground is relatively high, while the accuracy of the model of the middle scene is moderate, otherwise, the model of the long-range is relatively low, and even can be expressed by the way of map mask or image substitution, so that the virtual reality can be optimized in real time according to the different perspectives of the scene.

### 3.2. System of Face Tracker

The main task of face tracker is to determine the size, position, distance and other attributes of facial features such as iris, nose wing, mouth corner and so on, and then their geometric features are calculated to form a feature vector to describe the face as a whole [24]. The core principle of the technology is to follow the analysis of local human feature and algorithm of neural recognition. The main purpose of this paper is to compare, judge and confirm all the original parameters in the recognition database based on the features of human facial activity.

### 3.3. System of Gesture Tracker

The system of gesture tracker is based on Oculus quest2 hand positioning and tracking technology, which can capture the spatial coordinates of the joints of human hands, and transmit them to the animation of virtual reality in real time [25]. The main principle is to collect the bending posture of each finger, and make all fingers form a data format of unified single byte through data normalization algorithm, so as to reduce redundant data. At the same time, smoothing algorithm is used to process the spatial and temporal parameters between fingers to make the skeleton and muscle of gesture form a natural and soft state [26].In addition, in the process of gesture capture, segmentation methods based on obvious features will be formed, including skin color segmentation and hand shape segmentation.

1. Skin-color segmentation: it is a method of using cluster skin color to establish skin color model in precise coordinates, which comprehensively confirms skin color with the help of RGB color gamut
2. Handshape segmentation: it is a method based on multi-mode integration, which is mainly to overcome the limitations of segmentation conditions of the main structure in complex environment, and improve the apparent characteristics and motion information of hand. The strategies that commonly used include segmentation of geometric features, deformable features and spatial coverage features.

### 3.4. Camera System

The camera system in virtual reality means the input of the first view angle, which is also a form of active vision calibration that can effectively record the dynamic scene observed by human eyes [27, 28]. Different from the traditional virtual camera, it does not need to use a calibrated object of known size, but establishes the coordinate points and image points on the calibration of object. If the access of stable camera function needs to be get, it is necessary that program optimization work must be completed at the bottom of the program.

## 4. Design of Music Teaching System Based on Virtual Reality Technology

### 4.1. Overall Design

Based on the analysis of the system principles above, it can be concluded that the ideas of virtual reality in music teaching should be studied from three-dimensional modeling, facial capture, gesture capture, camera processing and other aspects. Firstly, it is necessary to use 3dsmax as the initial tool to complete the modeling of scene and role. After all models are improved, the scene model and character model should be imported into platform of Unity3d virtual reality, and the model embedding system in the platform should be used to make appropriate geometric segmentation of the model, and determine the relationship between LOD of different levels and the scene [29]. Secondly, the system of face tracker is used to identify and bind the faces of singer, and manages the positioning points of the main structure. Thirdly, the nodes of hand bone are confirmed by system of gesture tracker, and the corresponding data are calculated simultaneously with the interface of virtual reality engine. Finally, by optimizing the camera system, the singer's performance can be recorded in real time, which is convenient for the follow-up to analyze and evaluate the changes before and after the application of virtual reality. Generally speaking, the process above is based on an efficient and concise idea, as shown in Figure 1.

### 4.2. Creation and Optimization of Model

Model is very important in the process of production and experience. The structure accuracy and patch distribution of the model will directly affect the degree of simulation and interaction of virtual reality.

#### 4.2.1. Creation of Model

*(1) Scene Model*. Taking a scene of T-shaped stage as an example, the main methods are as follows:

1. First, use spline in 3dsMax to create a T-shaped stage of 3000 cm (length) × 2200 cm (width) × 1000 cm (height), convert it to polygon edit, and weld each vertex into a whole, so as to facilitate the subsequent connections of each boundary.
2. Secondly, use grid wiring to process the details of the overall model, with functions such as connection, extrusion, chamfering, and insertion to refine the local structure of the stage model. After independent modeling, the overall bridge is carried out.
3. Finally, use geometric lofting and polygon editing to create auxiliary models such as auditoriums and top light stands around the stage. During the modeling process, mirroring and copying of simple models can be used to enrich the overall scene, such as Figure 2.

*(2) Role Model*. The role model should be created under box elements, while the face and body of the role should be wired as a whole with polygon editing. It is necessary to ensure the wiring of facial features, body joints and other areas that need movement under virtual reality animation, and refine the structural relationship. In some areas that do not participate in animation motion, the number of model faces can be effectively controlled by means of collapse, patch merge, etc. which is shown in Figure 3. The unavoidable triangular wiring in the model is placed in the hidden area where the character does not participate in the animation calculation, so as to avoid the unfavorable phenomena such as patch folds in the animation of virtual reality.

#### 4.2.2. Optimization of the Model

In this process, the model is imported as a whole into Unity3D, the frame rate of the preview virtual reality is setto 70∼90 FPS, and the vertex closures of the model patches is deleted in the engine. In addition, the code is implanted at the blueprint interface where secondary optimization of the subtle parts of the scene is carried out. In order to meet the optimization of geometric segmentation, spatial coordinates, patch processing, rendering baking and other aspects of the model, the program design is as follows:

  int main (int, char^*∗∗*^) {
  osg Producer:: Viewer viewer; &par; Create a scene
  viewer. set UPViewer ( ) ：
  II Load the osga terrain model into the node variable
  osg:: Node ^*∗*^ node = osg DB::read Nodefile (“Wutai. osga”):
  viewer.set Scene Data(node); II Load the model into the scene
  &par; Enter the rendering loop
  viewer. realize ( );
  while (! viewer. done ( ) ) {
  viewer.sync( ); II Wait for the completion of all cull and draw threads
  viewer.update( ); II Update the scene by traversing the nodes
  viewer.frame( );&par;Render the updated result
  }
  viewer.sync( ); II Wait for the completion of all cull and draw threads before exiting the program
  return;
  }

### 4.3. Capture of the Face

Due to the principle of structured light adopted by the system, it is necessary to project light in the direction of the face, and then use the data that is on the surface of the object to be read to determine the shape of the face [30]. When choosing a face acquisition device, in addition to configure distance sensors, microphones, and front-facing cameras, it is also necessary to have infrared lenses, floodlights, floodlight sensing elements and dot matrix projectors arranged in sequence. Usually, the dot projector can project a dot matrix composed of more than 30,000 invisible light points to the face, then the face captured by the front-facing camera is simultaneously calculated to obtain the depth information of the facial expression, that is, the 3D model of real face. The four data interfaces that need to be built for simultaneous calculation are as follows:

- 1IFTFace Tracker: the main interface for face tracking.
- IFTResult: the result of face tracking.
- IFTImage: image buffer.
- IFTModel: model of 3D face.
- The data that needs to be acquired in simultaneous calculation are as follows:
- FT_CAMERA_CONFIG: color or depth sensor data.
- FT_VECTOR2D: two-dimensional vector data.
- FT_VECTOR3D: 3D vector data.
- FT_ Translate (XYZ): all input data required for face tracking.
- FT_Rotate(*X* Y *Z*): 3D model of face angle data.
- FT_Scale(*X* Y Z): weight matrix data, as shown in Figure 4.

Compared with methods of face tracker, The accuracy of face recognition of *T*_*j*_ is 0.1 mm, which can exceed image 2, video 1mmc1and plane 0. When light conditions of *R*_*i*_ is not ideal, the method of obtaining facial information, such as the light -*σ* and the received light *s* emitted by the dot projector will not affect the recognition efficiency of *T*_*j*_, whose system of face tracker can be changed as follows:

(1) $$\begin{array}{c} T_{j}\left(x,y\right)=\left\{\begin{array}{cc} 2 & if\;R_{i}\left(x,y\right)<-\sigma \\ 1 & if\;R_{i}\left(x,y\right)>\sigma \\ 0 & if\;-\sigma \leq R_{i}\left(x,y\right)\leq \sigma \end{array}\right). \end{array}$$

### 4.4. Capture of Gestures

Capture of gestures is a technical difficulty in virtual reality, which needs to be connected to the computer through the singer wearing a virtual head-mounted display device “Oculus quest2” and a hand tracker. After that, a depth-sensing camera is installed at the front of the head-mounted device and tilted downward by 13.4°, so that the singer can observe his hands in real time during the experience of virtual reality and track the changes of their fingertips in time. The gestures from left to right are: backward, stop, forward. If the position of the fingertip is within the zero-coordinate static zone (zc), no movement can be produced; However, when the fingertip extends forward beyond the static zone, the red progress bar of the subject's movement speed will increase linearly with the distance of the fingertip; In addition, when the finger joints move in the other direction and faces the palm downwards, the red progress bar will produce a subtle movement backwards. Specifically, it is a process of natural expansion and contraction of the palm. The process is based on the distance from the far end of the index finger of the singer's right hand to the center of the palm, and is proportionally enlarged by 2.74 times according to the size of each person's palm, so as to reduce the bending of the fingers. The noise caused by its setting parameters are as follows:

1. *β*: beta coefficient, *β* represents slope coefficient = velocity/*γ* (the distance from the index fingertip to the boundary of the static zone), forward movement *γ* = (position × 2.74)-(zc + dzw), backward movement *γ* =(zc-dzw)-(position × 2.74).
2. Dead zone: at the beginning of the test, the testers put their hands in a relaxed and gently bent position. Then, the zero rest position of the gesture can be determined when their fingers are in a comfortable position, as shown in Figure 5.
3. *α*: exponent-velocity = (*β* × *γ*)^*α*, when one parameter changes, the other parameters are fixed at their intermediate values. For example, *β* = 21 m/s, dzw = 25 mm, *α* = 1.0. The order of the three parameters is coefficient, static zone width, and exponent *α*, which was randomized. For each parameter, participants completed a large (2m) experiment (30 goals) and a small (1m) experiment (30 goals), while the order between these three parameters is not random.

In this experiment, it is required to complete the last 24 of the 30 indicators at least. Repeated measurement was used to analyze the differences of time at diverse levels, so as to separate the details of small targets and large targets. The settings are shown in Tables 1 and 2.

### 4.5. Establishment of Multiview Camera

In order to better improve the stability of the camera in virtual reality, and to enable the singers to examine the comprehensive performance of their actions and facial expressions in the virtual space from angles of multiple camera, it is necessary to optimize the bottom layer of the program., the code is modified as follows:

  Camera _camera;
(i) II Use this for initialization
(ii) void Start ( )
  {
  _camera = Camera.main;
  }
  IIThe first 3 locks of unity, from low to high are nothing/everything/default/transparent FX/ignore raycast/water UI
(iii) From the 1st to the 3rd can be set optional
  II The first is the cube layer; the second is the sphere layer; and the third is the capsule layer
  void Update ( )
  {
  if (Input.Get Key Down (Key code.A) )
  {
  _camera.culling Mask = 1 < < 1; ||cube, only render the first one
  }
  if (Input. Get Key Down (Key Code. B) )
  {
  _camera.culling Mask = 1 <<2; ||sphere, only render the second one
  }
  if (Input.Get Key Down (Key Code.S))
  {
  _camera.culling Mask = 1<<3; ||capsule, only render the 3rd one}

Through the method above, it can be observed that the stability of the multi-view camera is ideal, which is convenient for subsequent quantitative analysis of the singer's performance, as shown in Figure 6.

### 4.6. Evaluation of the Test

Subjects: 20 students majoring in vocal performance, 10 males and 10 females each, 5 people per time, who are divided into 4 groups according to the groups and gender. Virtual content: the content of the custom-made 360° virtual vocal video is divided into 6 songs according to emotional classification: positive (excited), neutral (comfortable), and negative (sad), which are respectively: positive emotional songs “My Motherland and Me,” “On the Field of Hope,” negative emotional songs “Where Has Time Gone,” “Mother in Candlelight,” neutral emotional songs “Baykal Lake” and “Pastoral.”

Experimental results: The data collection and analysis were carried out in the form of questionnaires and SAM, and the results were good, as shown in Table 3.

The high-fidelity vocal interaction was obtained through the SAM, and the corresponding analysis was made before and after intervention of virtual reality, as shown in Figure 7.

From the analysis of the scale data, it can be seen that the emotional changes produced by the use of the high-fidelity vocal interactive virtual system are much higher than the traditional music teaching, which is mainly due to the immersion and high simulation brought by virtual reality technology.

## 5. The Application Prospect of Virtual Reality Technology in Music Teaching

When VR is applied in education, students can be more focused and more active. This advantage comes from the immersion of VR itself, which cannot be provided by traditional teaching methods. In the teaching process of VR, students can have a higher degree of participation and better integrate into the whole process [31, 32]. For subjects that require a certain amount of imagination, virtual reality technology can simulate some scenes that cannot be realized in ordinary class from diverse directions.

The virtual realization of music works and courses is mainly constructed through 3D animation and 3D roaming. In actual production, software such as 3DMAX and Unity3d is used to create multiple virtual scenes such as oceans, deserts, grasslands, forests, European castles and then they are placed in the module with different styles of music. After students enter the module and select the corresponding virtual scene, the music will be played together, which allows students to experience the music in combination with the environment. Moreover, it creates an immersive feeling and realizes situational teaching. For example, in the teaching of folk songs, students can enter the virtual scene of forests, mountains and rivers, and feel the charm of songs immersively.

Through the application of virtual reality technology, users can feel like entering a real concert hall or music classroom. That is to say, when users employ the virtual experience module, they can use the mouse to click and select different positions on the interface. Through the user's click and selection, the interface is displayed in a three-dimensional manner, which let the experiencer have an immersive feeling. The specific content of the virtual experience can be set according to the actual teaching of different majors. During the development of the system, many data interfaces are reserved, and the text, background music, pictures and other contents of the experience hall can be set according to the teaching tasks of different majors.

The analysis of functional module can be designed with students' major in music production as the main object, in which the effect of actual works of art is taken as an example. Detailed explanation and elaboration of the professional techniques and principles used in the works is received, and in this way, the effect of virtual reality is fully utilized to make the corresponding class more vivid, which provides students a better interactive experience. In musical instrument teaching, students can check the performance from different angles, which is almost the same as the effect of live teaching. Others, such as classical music and vocal music, also have the same advantages for teaching in the application.

The interaction model is the main functional module of learning and resource sharing. This function needs to provide the Unity 3D default plug-in, which is implemented by self-coding. The rotation angle range is calculated by moving the distance of the mouse, and the angle of view is controlled by Clamp Angle to complete the calculation of the angle. Then according to the relative distance between the camera and the object, the relative coordinates of the camera are calculated, and values are assigned, finally the setting of the entire camera position and angle parameters are completed to ensure the effectiveness of the perspective interaction.

## 6. Conclusion

In the process of education and teaching, virtual reality technology can realize interactive teaching through human-computer interaction, which brings convenience to teachers and students, and prompts the birth of a new teaching mode. Due to the limitations of musical equipment, conventional music teaching is carried out in a relatively enclosed environment, and its guidance is implemented one-on-one by teachers. In particular, courses such as vocal music, piano, and instrumental music performance usually require students to “feel with their hearts”, which is highly subjective. The infinite extensibility and abundant teaching expressiveness of virtual reality interactive teaching can make the teaching more attractive. Moreover, using information technology to integrate virtual reality technology into music teaching, as well as building a specific place in an abstract way to provide students a “realistic” learning environment, can stimulate students' autonomous learning it.

## Figures and Tables

**Figure 1:** Design of work flow.

**Figure 2:** Model of Stage scene.

**Figure 3:** Role model.

**Figure 4:** The effect after facial capture.

**Figure 5:** Zero stillness of gesture.

**Figure 6:** Effect of multi-view camera.

**Figure 7:** Comparison before and after the intervention of virtual reality.

**Table 1:** Beta coefficient (small target) (m/s).

	*β* = 12	*β* = 21	*β* = 30	*P* value
Total time (s)	74.5 (48.0)	62.6 (18.3)	82.0 (31.4)	0.18
Excellent control	4.5 (0.5)	3.8 (0.9)	3.6 (0.7)	0.0001
No shoulder fatigue	4.2 (0.9)	4.1 (1.0)	4.2 (1.1)	0.65

**Table 2:** Dead zone width (small target) (mm).

	dzw = 10	dzw = 25	dzw = 40	*P* value
Total time (s)	71.9 (22.8)	71.0 (32.5)	73.0 (38.2)	0.94
Excellent control	3.5 (0.7)	3.8 (0.9)	4.2 (0.9)	0.15
No shoulder fatigue	4.4 (1.0)	4.2 (0.9)	4.3 (1.0)	0.59

**Table 3:** Data analysis of the experience of using the vocal interactive virtual system.

Index	Excellent (%)	Good (%)	Generally (%)	Poor (%)
Immersive experience	90	10	0	0
Intelligent interaction	95	5	0	0
Fluency	99	1	0	0
Module completeness	80	15	5	0

## Data Availability

The dataset can be accessed upon request.
